RETRACTED

# Association of Pentachlorophenol with Fetal Risk of Prolonged Bradycardia: A Systematic Review and Meta-Analysis

**DOI:** 10.1155/2022/7552294

**Published:** 2022-03-27

**Authors:** Xueyun Song, Xiaodong Fu

**Affiliations:** Department of Obstetrics, The Affiliated Hospital of Southwest Medical University, Luzhou, Sichuan Province, China

## Abstract

**Objective:**

This study explored the systematic evaluation and meta-analysis of different concentrations of PCP on the risk of long-term bradycardia in fetuses.

**Methods:**

Cochrane Library, Embase, PubMed, China Biomedical Literature Service, CNCNKI, and Wanfang database were computerized to collect all case-control studies on the association between variety classes and different concentrations of environmental pollutant gas to fetal of prolonged bradycardia. After evaluating the quality of the inclusion study and extracting valid data, meta-analysis was performed using Stata15 software. Relative hazards were calculated using the Mantel-Haenszel method and the random effect model, and *P* values and *I*^2^ values were used for heterogeneity evaluation. When heterogeneity occurs, subgroup analysis and sensitivity analysis were used to explore the sources.

**Results:**

A total of 15 studies were included, including 1202 patients with fetal of prolonged bradycardia and 1380 in the control population. Meta-analysis showed that there was no statistical difference in PCP < 0.1 mg/L between the experimental group and control group (OR = 1.03, 95% CI (0.62, 1.72), *P*=0.90, *I*^2^ = 0%, *Z* = 0.13), but there was a statistical difference in PCP > 5 mg/L (OR = 1.73, 95% CI (1.15, 2.58), *P*=0.008, *I*^2^ = 0%, *Z* = 2.65), PCP > 10 mg/L (OR = 1.75, 95% CI (1.19, 2.57), *P*=0.004, *I*^2^ = 14%, *Z* = 2.85), and PCP >15 mg/L (OR = 2.02, 95% CI (1.38, 2.95), *P*=0.0003, *I*^2^ = 77%, *Z* = 3.61).

**Conclusion:**

In this study, we found that different concentrations of PCP increased the risk of long-term bradycardia in fetuses, and the risk coefficient increased with the increase of PCP concentration.

## 1. Introduction

Fetal bradycardia was defined as a fetal heart rate below 110 beats/min and with a duration longer than 10 min. The transient decline in fetal heart rate in middle and late pregnancies recovered in a short period of time and had a good prognosis [1]. Pathologic changes, such as sinus bradycardia, atrioventricular block, and long QT syndrome, should be considered when the fetal bradycardia continues. Persistent bradycardia is not common, accounting for about 5% of fetal arrhythmias, and can occur during various periods of the fetus [2]. The main disease accounts for about 14%, including atrioventricular septal defect, left atrial heterogeneous, and large artery abnormalities [3]. Abnormalities of these structures can cause interference with the electrophysiological continuity between the fetal atrium and ventricles, leading to arrhythmias. Fetuses combined with cardiac anatomical abnormalities have a relatively poor prognosis [4, 5].

RETRACTED

Pentachlorophenol (PCP) is a white needle crystal, highly volatile, heated when irritant phenol odor, hardly soluble in water, and easy to be soluble in ether, acetone, benzene, and other organic solvents. Pentachlorophenol is widely used as pesticides, antibiotics, and preservatives, covering industrial and commerce, agriculture, water industry, and home life. Due to its high toxicity, long persistence, and difficult degradation, its extensive use and improper treatment lead to the pollution of soil and water resources and has become an environmental pollutant that cannot be ignored [6]. PCP and Na-PCP are slowly degraded in natural environments. It can be enriched in the bottom mud, and the long-term heavy use has caused environmental pollution and biological accumulation. Although many countries, including China, have banned the continued use of PCP, its residual effect will last for years or even decades [7]. A certain level of trichlorophenol can be detected in the water bodies, soil, and plants in the contaminated areas. Pentachlorophenol can have toxic and a series of adverse effects through direct contact (skin and respiratory tract) or food chain enrichment. Pentachlorophenol into the human body can accumulate in the liver, kidney, and adipose tissue for a long time, produce toxicity to the liver and kidney, improve the incidence of tumor, interfere with endocrine, affect immune function, and hinder reproductive development. Pentachlorophenol is not only a direct hazard to the human body, but may be potentially dangerous to electrophysiological function of fetal heart [8].

PCP has a strong uncoupling effect and can cause acute or chronic poisoning in humans and animals. In recent years, numerous studies have shown that PCP contains highly toxic dibenzene dioxin (PcDDs), tetrachloride diphenylfuran (TcBDFs), and other pollutants, especially the highly toxic tetrachlorodibenzene dioxin (TCDD). These substances have strong carcinogenic, teratogenic, mutagenic effects, with a greater impact on the reproductive system. Based on their strong biological stability, they will also be stronger and more durable. In addition, PCP has a strong adsorption to the soil and sediment; PCP water source irrigated crops will affect product quality; fishery will cause pollution to the environment of aquaculture waters, affect the healthy growth of fish, or cause death [9]. In the areas where PCP was used, the produced food PCP content, human daily intake, and urinary PCP concentration were significantly higher than that of the control region. After PCP enters the human body, it circulates to the tissues and organs of the whole body, most of which are discharged from the urine, and about 20% can accumulate in the body. Relevant investigation shows that the content of PCP in residents in polluted areas is significantly increased compared with the control area; therefore, attention should be paid to the potential health harm of food residual PCP to human body [10].

RETRACTED

Although the use of PCP has been banned in China, its residual effect will persist for a long time; Na-PCP is still the best and cheapest sterilization effect in China, and this study was to explore the effects of different concentrations of environmental pollutants (PCP) on fetal bradycardia.

## 2. Materials and Methods

### 2.1. Search Strategy

Medline, Embase, Cochrane CENTRAL, Chinese Journal Full Text Database (CNKI), Chinese Biomedical Database (CBM), Chinese Science and Technology Journal Full Text Database (VIP), and Wanfang database were searched by computer. Manual retrieval of references is to important literature. Key search terms: “Environmental pollutant,” “Fetal bradycardia,” “Fetal arrhythmia,” and “Fetal prognosis”. All databases were searched from October 2000 to October 2021.

### 2.2. Literature Selection Criteria

1. Inclusion criteria: all studies related to fetal bradycardia and environmental pollutants were selected in strict accordance with PRISMA statement, provide data on fetal arrhythmia and concentrations of targeted environmental pollutants, provide sufficient data to calculate OR and 95% CI, case-control study, get full text, duplicate publications from the same population were used, and the largest sample size was selected for inclusion in the study.
2. Exclusion criteria: incomplete data, studies, case reports, reviews, reviews, summaries, and basic research based on pedigree data.

### 2.3. Data Extraction and Processing

Two researchers used a unified data extraction table to extract data independently and then cross-checked the data. If necessary, they contacted the authors of the original literature to determine the specific implementation process of the experiment. According to inclusion criteria, the following information was included: first author, year of publication, region, ethnicity, type of arrhythmia (fetal bradycardia and tachycardia), environmental contaminants and concentration detection methods, total number of cases, control group, study quality score, and cases. If two researchers have a dispute during data extraction, a third researcher will help resolve the discussion after referring to the original text.

RETRACTED

### 2.4. Quality Evaluation of the Included Study

There are 3 researchers who independently evaluated the study based on a quality assessment form developed in the prior study quality. The score ranges from 0 to 13, with 0 being the lowest quality and 12 being the highest quality (Figure 1).

### 2.5. Bias Analysis

Heterogeneity between studies was assessed using *I*^2^ statistics, and 25%, 50%, and 75% representing low, medium, and high heterogeneities, respectively; if *I*^2^ 50% and *P* > 0.1 between studies using fixed-effect models and if *I*^2^ > 50% and *P* < 0.1 from chi-square analysis showed study heterogeneity, meta-analysis is by random effects models and searched for possible heterogeneity by subgroup analysis source. The sensitivity analysis removed the included literature one by one to see whether the pooled effect values were stable and reliable (Figure 2).

### 2.6. Statistical Analysis

RevMan 5.2 statistical software was used for meta-analysis. Heterogeneity was assessed by the *t*-test at a significant level *α* = 0.10 (*P* < 0.1 or *I*^2^ > 50%). The results without heterogeneity were combined and analyzed by the fixed-effect model, while those with heterogeneity were analyzed by the random effect model. Mean difference (MD) and its 95% confidence interval (CI) combined effect were used for continuous variables with the same measurement units, and relative risk (RR) and its 95% CI combined effect were used for categorical variables.

## 3. Result

### 3.1. Retrieving the Results and Incorporating Basic Information in the Study

359 literatures were obtained according to the retrieval strategy, and the remaining 108 literature entered the screening process after the exclusion of duplicate literature. 15 articles were selected for preliminary screening, among which two English articles were excluded due to lack of reported inclusion outcome indicators. 15 articles were finally included, with a total of 1397 patients [11–25]. There were 864 cases in the experimental group and 533 cases in the control group (Figure 3). Basic information of included studies is given in Table 1.

### 3.2. PCP < 0.1 mg/L

Among the 4 RCTs literature included in environmental pollutant concentrations with fetal risk of prolonged bradycardia, the heterogeneity test was carried out, and it was found that the heterogeneity of the selected studies was small, so meta-analysis with fixed models could be performed. Meta-analysis results showed that there was no statistical difference in PCP < 0.1 mg/L between the experimental group and control group (OR = 1.03, 95% CI (0.62, 1.72), *P*=0.90, *I*^2^ = 0%, *Z* = 0.13) (Figure 4).

RETRACTED

### 3.3. PCP > 5 mg/L

Among the 4 RCTs literature included in environmental pollutant concentrations with fetal risk of prolonged bradycardia, the heterogeneity test was carried out, and it was found that the heterogeneity of the selected studies was small, so meta-analysis with fixed models could be performed. Meta-analysis results showed that there was a statistical difference in PCP > 5 mg/L between the experimental group and control group (OR = 1.73, 95% CI (1.15, 2.58), *P*=0.008, *I*^2^ = 0%, *Z* = 2.65) (Figure 5).

### 3.4. PCP > 10 mg/L

Among the 4 RCTs literature included in environmental pollutant concentrations with fetal risk of prolonged bradycardia, the heterogeneity test was carried out, and it was found that the heterogeneity of the selected studies was small, so meta-analysis with fixed models could be performed. Meta-analysis results showed that there was a statistical difference in PCP > 10 mg/L between experimental the group and the control group (OR = 1.75, 95% CI (1.19, 2.57), *P*=0.004, *I*^2^ = 14%, *Z* = 2.85) (Figure 6).

### 3.5. PCP > 15 mg/L

Among the 4 RCTs literature included in environmental pollutant concentrations with fetal risk of prolonged bradycardia, the heterogeneity test was carried out, and it was found that the heterogeneity of the selected studies was small, so meta-analysis with fixed models could be performed. Meta-analysis results showed that there was a statistical difference in PCP > 15 mg/L between the experimental group and control group (OR = 2.02, 95% CI (1.38, 2.95), *P*=0.0003, *I*^2^ = 77%, *Z* = 3.61) (Figure 7).

## 4. Discussion

PCP in the environment mainly comes from the production and improper processing of the product. It is reported to produce 2,000 tPCP or Na-PCP, and the exhaust gas will contain 18tPCP, 9 t of other phenolic compounds. Na-PCP produces large amounts of PCP and other phenol wastewater; PCP can also be discharged directly into the environment by related industrial wastewater [26]. PCP-treated wood is also being released directly into the environment when used or burning.

Many animal experiments have confirmed that PCP has certain reproductive toxicity to organisms. For example, PCP can inhibit the growth and development of hamster oocytes; cows fed containing PCP found pathological changes such as luteal insufficiency and abnormal oocyte development [27]. After sexual maturation, ranging from 7 to 8 d, both the proportion of female mink receiving the second mating and the rate of lactation was decreased. R raised with feed containing PCP and necrolysis from the beginning of embryonic stage to week 28, the preferential margin of the scrotum increased, and the atrophy of the semen tube increased. The epididymal sperm density was decreased. In 2002, Bemard et al. fed 2 generations of SD rats with PCP, and reproductive toxicity tests showed that high-dose (60 mg/(kg.d)) feeding caused delayed sexual maturation, reduced sperm number, reduced prostate and testes, reduced embryo implantation capacity, and reduced litter production [28].

RETRACTED

Similarly, in humans, with the deterioration of environmental quality, many environmental pollutants can pass through the way such as respiratory tract, the digestive tract, the skin into pregnant woman's body, and then through the limited tire barrier into fetal body because the fetus is sensitive to the chemical poison effect than adults; in the process of growth and development, if some poisonous substances contact within the womb, it may produce some effects, and adult contact with the substance is not the same as severe damage or even cancer [29, 30].

PCP is an anticompetitive inhibitor of human placental alkaline phosphatase (PLAP). Toxicology tests show that PCP is a strong mitochondrial unconjugation agent that reduces plasma membrane mobility and also has a strong inhibitory effect in the acetylcholinesterase on the cell membrane [29]. Placental alkaline phosphatase is a metalloglycoprotein located on the membrane of late placental cells; in addition to catalytic function, some substances such as IgG, complement factor B, and cartilage matrix protein are related to fetal growth and development. Changes in the PLAP conformation can not only alter its function but also cause the structure and function of the placental cell membrane change, which must have adverse effects on the normal fetal development. In addition, PCP is a lipid-soluble substance that can enter the fetus through the placenta and have a direct toxic effect on the fetus [30]. In Heidelberg Hospital, Germany, during a physical examination of 65 women with a long history of PCP exposure, it was found that its serum PCP content was asked above 20 bucket g/L; thus, the exposure history of PCP in pregnant women will also have adverse effects on the fetus.

Fetal arrhythmias caused by the toxic effect of PCP are common in routine prenatal ultrasound screening and can occur throughout any stage of pregnancy, with the incidence reported in foreign literature during pregnancy of up to 1–3%. Fetal JbL, arrhythmias can be divided into three categories: irregular arrhythmias, tachycardia, and bradycardia, among which irregular arrhythmias are the most common, mainly caused by prephase contraction. The most common fetal tachycardia is intraventricular tachycardia and atrial fibrillation. The most common fetal bradycardia is complete atrioventricular block; the mother of children is with normal heart structure. There are high-efficiency anti-SSA antibodies or anti-SSB antibodies staring inside.

RETRACTED

The limitations of this study are as follows: incorporating observational studies in the study is limited, the follow-up varies from 3 to 36 months, making the evaluation of long-term complications, the publication bias analysis is only qualitative and large personal factors, and the two techniques described in this study contain multiple surgical procedures, which may increase the bias of the article. Since the assessments were all based on a small number of studies [26–28], the results must be interpreted with caution. As the accumulated evidence grows, our conclusions may either be supported or overturned.

## 5. Conclusion

In conclusion, environmental pollutant PCP > 0.1 mg/L could increase the risk of fetal bradycardia, and it increased with the increase of PCP concentration. It is of great significance to evaluate the toxic effects of maternal exposure to environmental pollutants in order to reduce the health damage to the next generation.

## Figures and Tables

**Figure 1:** Literature quality evaluation chart. (a) Risk of bias graph. (b) Risk of bias summary.

**Figure 2:** Funnel plot of literature publication bias for PCP < 0.1 mg/L (a), PCP > 5 mg/L (b), PCP > 10 mg/L (c), and PCP > 5 mg/L (d) between two groups.

**Figure 3:** Flowchart of the literature screening.

**Figure 4:** Meta-analysis of PCP < 0.1 mg/L between two groups.

**Figure 5:** Meta-analysis of PCP > 5 mg/L between two groups.

**Figure 6:** Meta-analysis of PCP > 10 mg/L between two groups.

**Figure 7:** Meta-analysis of PCP > 15 mg/L between two groups.

**Table 1:** Basic clinical features of 15 literature were included in our study.

Study	Pregnant time (W)	Environmental pollutant	Experimental group (*N*)	Control group (*N*)	NOS score	Research type	*P* values
Kállay K, 2019	23.71 ± 2.2	Pentachlorophenol (PCP)	96	75	8	RCT	0.35
Duffy C, 2019	25.65 ± 3.4	Pentachlorophenol (PCP)	86	63	8	RCT	0.02
Lei H, 2020	32.12 ± 4.5	Pentachlorophenol (PCP)	118	108	8	RCT	0.04
Holmberg, 2020	27.15 ± 4.5	Pentachlorophenol (PCP)	66	60	7	RCT	0.12
Khera R, 2019	32.45 ± 3.4	Pentachlorophenol (PCP)	58	73	8	RCT	0.06
Gálvez JA, 2019	24.26 ± 1.2	Pentachlorophenol (PCP)	54	65	7	RCT	0.02
Bush B, 2018	32.45 ± 2.2	Pentachlorophenol (PCP)	80	75	9	RCT	0.01
Rau C, 2021	32.51 ± 3.0	Pentachlorophenol (PCP)	80	63	8	RCT	0.02
Zhang B, 2020	27.25 ± 4.5	Pentachlorophenol (PCP)	41	56	7	RCT	0.14
Jamal A, 2020	26.22 ± 5.2	Pentachlorophenol (PCP)	64	70	8	RCT	0.23
Mamsen, 2019	31.35 ± 2.1	Pentachlorophenol (PCP)	108	100	7	RCT	0.01
Sol CM, 2020	27.65 ± 6.0	Pentachlorophenol (PCP)	96	77	7	RCT	0.25
Pan Y, 2020	25.65 ± 2.2	Pentachlorophenol (PCP)	22	25	8	RCT	0.14
Rokoff LB, 2018	24.62 ± 3.5	Pentachlorophenol (PCP)	44	32	8	RCT	0.07
Eladak S, 2018	31.46 ± 2.0	Pentachlorophenol (PCP)	25	30	8	RCT	0.35

RETRACTED

## Data Availability

The data used to support this study are available from the corresponding author upon request.
